The article "Zinc biofortification potential of diverse mungbean [Vigna radiata (L.) Wilczek] genotypes under field conditions" was retracted in 2022. Reasons: compromised peer review; a conflict of interest; concerns about the authorship.

# Zinc biofortification potential of diverse mungbean [*Vigna radiata* (L.) Wilczek] genotypes under field conditions

**DOI:** 10.1371/journal.pone.0253085

**Published:** 2021-06-23

**Authors:** Muhammad Umar Haider, Mubshar Hussain, Muhammad Farooq, Sami Ul-Allah, Mohammad Javed Ansari, Mona S. Alwahibi, Shahid Farooq

**Affiliations:** 1 Department of Agronomy, Bahauddin Zakariya University, Multan, Pakistan; 2 Department of Crop Sciences, College of Agricultural and Marine Sciences, Sultan Qaboos University, Al-Khoud, Oman; 3 Department of Agronomy, University of Agriculture, Faisalabad, Pakistan; 4 College of Agriculture, Bahauddin Zakariya University, Layyah, Pakistan; 5 Department of Botany, Hindu College Moradabad, Mahatma Jyotiba Phule Rohilkhand University, Bareilly, India; 6 Department of Botany and Microbiology, College of Science, King Saud University, Riyadh, Saudi Arabia; 7 Departmnet of Agronomy, Faculty of Agricultural Sciences, Ghazi University, Dera Ghazi Khan, Pakistan; Government College University Faisalabad, PAKISTAN

## Abstract

Zinc (Zn) is an important micronutrient for crop plants and essential for human health. The Zn-deficiency is an important malnutrition problem known globally. Biofortified foods could overcome Zn deficiency in humans. Mungbean [*Vigna radiata* (L.) Wilczek] is an important, pulse crop frequently grown in arid and semi-arid regions of the world. Mungbean could provide essential micronutrients, including Zn to humans. Therefore, it is very important to investigate the impact of Zn fertilization on the yield and grain biofortification of mungbean. Twelve mungbean genotypes (i.e., NM-28, NM-2011, NM-13-1, NM-2006, NM-51, NM-54, NM-19-19, NM-92, NM-121-25, NM-20-21, 7006, 7008) were assessed for their genetic diversity followed by Zn-biofortification, growth and yield under control (0 kg ha^-1^) and Zn-fertilized (10 kg ha^-1^) conditions. Data relating to allometric traits, yield components, grain yield and grain Zn contents were recorded. Zinc fertilization improved entire allometric and yield-related traits. Grain yield of different genotypes ranged from 439 to 904 kg ha^-1^ under control and 536 to 1462 kg ha^-1^ under Zn-fertilization. Zinc concentration in the grains varied from 15.50 to 45.60 mg kg^-1^ under control and 18.53 to 64.23 mg kg^-1^ under Zn-fertilized conditions. The tested genotypes differed in their Zn-biofortification potential. The highest and the lowest grain Zn contents were noted for genotypes NM-28 and NM-121-25, respectively. Significant variation in yield and Zn-biofortification indicated the potential for improvement in mungbean yield and grain Zn-biofortification. The genotypes NM-28 and NM-2006 could be used in breeding programs for improvement in grain Zn concentration due to their high Zn uptake potential. Nonetheless, all available genotypes in the country should be screened for their Zn-biofortification potential.

## Introduction

Mungbean [*Vigna radiata* (L.) Wilczek] is an important legume crop of arid and semi-arid regions in the world. It is moderately drought-tolerant; however, severe droughts exert negative impacts on its growth and production [1]. High edible protein contents in the seeds of mungbean make it an important and superior food legume. It has healthier digestible protein contents than other pulses grown worldwide [2]. Mungbean grains contain 3% fat, 3.5–4.5% fibers, 50% carbohydrates, 26% protein and 3% vitamins [3]. It is mostly grown in marginal and arid lands despite its importance in combating hidden hunger and alleviation of poverty.

Hidden hunger is a term used to describe micronutrients’ deficiency in humans. Zinc is an essential nutrient, absorbed in the form of divalent cations and important for plant growth and productivity [4]. It is a vital micronutrient for human health, as it is involved in numerous metabolic processes. Zinc-deficiency can cause serious health problems. Humans using Zn-deficit crops may suffer from several health issues, including retarded growth and development, stunted growth in children, susceptibility to diseases and meager immunity [5–7]. Deshpande [8] reported that Zn could decrease the severity and frequency of diarrhea in children. Moreover, adequate Zn intake is compulsory for the proper functioning of the immune system [8].

Pakistani soils are Zn-deficit, which not only leads to low Zn contents in edible parts of the crops, but also affects their growth and productivity [9, 10]. Zinc fertilization not only improves grain Zn concentration, but also important for the growth and productivity of mungbean [11, 12]. Nonetheless, the presence of Zn is necessary for the proper functioning of different plant systems, including nitrogen metabolism and protein synthesis [6, 13]. Furthermore, Zn plays an important role in the formation of chlorophyll and synthesis of carotenoids leading to better pollen formation, fertilization and photosynthesis [14–16]. The roles of Zn in the formation of stamens and pollen have recently been reported [17, 18], which improved the number of seeds per pod, reproductive branches and 1000-seed weight.

The provision of a Zn-enriched diet is a sustainable way to alleviate Zn-deficiency in humans. Pulses, especially mungbean, are an important part of the human diet throughout the world and a relatively cheap source of protein. Therefore, Zn-biofortification of mungbean is a viable option to combat Zn-deficiency. Various biofortification techniques include; improvement in Zn contents through breeding [6, 19], development of high Zn acquiring transgenic plants [20] and soil and foliar application of Zn [6, 19]. All these techniques improve Zn concentration in pulse grains; however, these methods are not equally efficient in all soil types and environmental conditions. Even in the same soil type and environmental conditions, genotypes respond differently to Zn-fertilization [19].

Recent studies have focused on the agronomic Zn biofortification of different crops such as mungbean and chickpea [21–24]. Zinc application through seed priming enhanced the growth, productivity and grain biofortification of chickpea [22, 23, 25, 26]. Similarly, Kanwal et al. [21] indicated that basal application of Zn improved productivity and profitability of mungbean. Recently seed priming [27, 28] and seed coating [29] have been used to improve the productivity and grain biofortification of mungbean. However, these studies used a limited number of genotypes.

Mungbean is frequently grown in semi-arid regions, marginal lands, monsoonal wet tropics and temperate regions. Furthermore, Zn fertilization is not a common practice in countries like Pakistan. Genotypes differ in their response to Zn biofortification; however, Pakistani mungbean genotypes have rarely been explored for their Zn-biofortification potential under field conditions. Therefore, this study evaluated genetically diverse mungbean genotypes for their grain Zn-biofortification potential and yield under Zn fertilization. The outcomes of this study will be important for both agronomists (for better mungbean production with high Zn contents) and plant breeders (for the development of Zn-biofortified, high-yielding mungbean cultivars).

## Materials and methods

### Experimental site and treatments

This study was conducted in the experimental area of the Department of Agronomy, Bahauddin Zakariya University, Multan, Pakistan (71.43^o^ E, 30.2^o^ N and altitude 122 m) during 2016. The site is located in a semi-arid region with a subtropical climate. Twelve genetically diverse mungbean genotypes were used to evaluate their grain Zn-biofortification potential under Zn (10 kg ha^-1^) and no-Zn (0 kg ha^-1^) treatments. The experiment consisted of two Zn levels (0 and 10 kg ha^-1^) and 12 mungbean genotypes (NM-28, NM-2011, NM-13-1, NM-2006, NM-51, NM-54, NM-92, NM-20-21, NM-19-19, NM-121-25, 7006 and 7008), which were obtained from Nuclear Institute for Agriculture & Biology (NIAB), Faisalabad, Pakistan. Commercially available zinc sulfate was used as Zn source and added to the soil during land preparation before sowing. The experimental soil was sandy loam with a pH of 8.1, 0.47% organic matter, EC of 2.39 dS m^-1^, 5.4 mg kg^-1^ P, 160 mg kg^-1^ K and 0.61 mg kg^-1^ Zn. The treatments were arranged in a randomized complete block design with split-plot arrangements. Genotypes were kept in main plots, whereas Zn treatments were randomized in sub-plots. The experiment had 3 replications. Net plot size was 1.8 m × 4 m where row × row and plant × plant distance was 45 and 20 cm, respectively. The field study did not require any permit and involved no endangered species.

### Genetic diversity analysis

For genetic diversity analysis, pure seeds of the tested genotypes were grown in polythene bags, fresh leaves (5 g) were taken from each genotype three weeks after emergence and washed with double sterile water to remove any contamination. After washing, the leaves were ground in mortar and pestle using a modified cetyl trimethylammonium bromide (CTAB) method following the standard protocol described by Englen and Kelley [30]. After DNA extraction, polymerase chain reaction (PCR) amplification was executed in a 20 μL volume reaction mixture. Ten ISSR markers were used for the amplification of DNA. The PCR reaction mixture consisted of 12.8 μL sterile deionized water (d2H_2_O), 1 μL DNA, 2.0 μL PCR buffer (10X), 0.5 μL 10 mM dNTPs, 2.5 μL MgCl_2_, 0.2 μL Taq Polymerase and 1.0 μL primer. The cycling conditions consisted of 5 min for initial denaturation at 95°C, 35 cycles of denaturation (1 min at 95°C), annealing (52°C for 1 min) and elongation (72°C for 2 min) followed by the final extension (72°C for 10 min), then cooled down to 4°C. The PCR products were injected with 2% agarose gel for visualization by gel electrophoresis.

### Crop husbandry

Before sowing, 100 mm pre-soaking irrigation was applied and the seedbed was prepared when soil moisture reached to field capacity level. Ridges were made with the help of a tractor-mounted ridger. Mungbean seeds were sown with dibbler using a seed rate of 20 kg ha^-1^ on June 7, 2016. Zinc sulfate was applied at 10 kg ha^-1^ with the help of a hand drill according to the treatments. The crop was irrigated regularly to avoid moisture stress. Fertilizers were applied at the rate of 30 and 80 kg ha^-1^ nitrogen and phosphorus, respectively using urea and triple superphosphate as sources. All agronomic management practices, including irrigation, fertilizer application and plant protection measures were done uniform for all the experimental units. Weeds were controlled manually. All the experimental units were harvested on the same day, i.e., September 29, 2016.

### Field data collection

For allometric traits, samples were collected by destructive method, i.e., an area of half-square meter was used to record root length, the number of lateral roots, dry weight of roots, leaves and stem, and leaf area per plant at 40, 55 and 70 days after sowing (DAS). The SPAD-502 chlorophyll meter was used to estimate the chlorophyll index (SPAD value) at 40 DAS. Data relating to morphological and yield-related traits plant height (cm), total number of pods per plant, pod length (cm), the average number of seeds/pod, total numbers of vegetative and reproductive branches) were collected at maturity from twenty plants and averaged. For the determination of grain yield (kg ha^-1^), two central rows from each plot were harvested at maturity, sundried until constant weight, weighed with the help of digital balance to record biological yield (kg ha^-1^) and threshed manually to record grain yield. Five samples of 1000 seeds were taken from each seed lot and weighed on an electric balance and averaged to record 1000-grain weight (g) according to Majeed et al. [31]. Grain yield was corrected to 10% moisture contents. Harvest index (%) was taken as the ratio of grain yield to the biological yield expressed in percentage.

### Grain Zn concentration

From each experimental unit, a 25 g grain sample was collected, grounded to pass from 1 mm sieve out of which 1 g was thoroughly mixed in 10 mL mixture (1:2 v/v) of 70% HClO_4_ and HNO_3_ in a Pyrex digestion flask and left overnight [32]. For digestion, the mixture was heated at 150°C until the production of red fumes stopped. After digestion, the mixture was kept at 250°C until the liquid became transparent. The volume of the sample was increased to 25 mL by adding distilled water and filtered. Atomic absorption spectrophotometer was used to estimate grain Zn contents (mg kg^-1^) following the procedure of Shobhana [33].

### Statistical analysis

Data collected from gel electrophoresis was scored in a binary fashion as 0 and 1 for the absence and presence of bands, respectively. The genetic diversity of the genotypes was assessed by grouping them based on the similarity index. Unweighted Pair Group Method with Arithmetic Mean (UPGMA) was executed using NTSYS-PC v. 2.0 software. Grain yield, yield components and Zn uptake data were analyzed using analysis of variance technique (F test) and treatment means were compared by the least significant difference test (LSD) at a 5% probability level [34]. Data were tested for normality by the Shapiro-Wilk normality test [35] before analysis, which indicated a normal distribution. Therefore, original, non-transformed data were used in the statistical analysis. For a graphical representation of data, Microsoft Excel software version 2010 was used.

## Results

### Genetic diversity

Molecular data showed significant genetic diversity among tested mungbean genotypes. Dendrogram divided the genotypes into nine subpopulations with a similarity index ranging from 0.82 to 1.0. The genotypes 7006 and NM-2006 were in the same group with a similarity index of 1.0. Similarly, the genotypes NM-92, NM-121-25 and NM-20-21 were in the same group with a similarity index of 1.0. All other genotypes had a <1.0 similarity index (Fig 1).

**Fig 1:** Dendrogram of mungbean genotypes based on the ISSR marker showing the genetic diversity and similarity index.

### Allometric traits

Allometric data (Figs 2 and 3) showed that the number of lateral roots and root length gradually increased with the life cycle of the crop, and Zn application improved all root traits compared with no-Zn application. The number of lateral roots and root length improved for all the genotypes with Zn application and the highest root length was recorded for genotype NM-54 and the lowest root length was noted for NM-2011. In the case of lateral roots, the highest number was observed for the genotype 7006 and the lowest was recorded for NM-121-25 (Figs 2 and 3).

**Fig 2:** Root length of various mungbean genotypes at various growth stages as affected by Zn fertilization.

**Fig 3:** Number of lateral roots of various mungbean genotypes at various growth stages as affected by Zn fertilization.

Periodic data showed improvement in leaf area index (LAI) up to 55 DAS followed by a decline due to leaf senescence at maturity; however, leaf area duration (LAD) increased until the last reading (Figs 4 and 5). Regarding genotypes’ performance, the trend of LAI and LAD remained the same. Genotypes sown with Zn application remained superior with higher LAI and LAD than the genotypes sown under no-Zn application (Figs 4 and 5). Among all genotypes, NM-92 and NM-51 observed the highest LAI and LAD, whereas the lowest LAI and LAD were recorded for genotypes NM-2011 and NM-20-21 (Figs 4 and 5).

**Fig 4:** Leaf area index of various mungbean genotypes at various growth stages as affected by Zn fertilization.

**Fig 5:** Leaf area duration of various mungbean genotypes at various growth stages as affected by Zn fertilization.

Periodic data showed improvement in the net assimilation rate (NAR) and crop growth rate (CGR) from 40 to 70 DAS (Figs 6 and 7). Genotypes sown with Zn application recorded higher CGR and NAR as compared to genotypes under control. The highest CGR was recorded for genotype NM-92, whereas the least CGR was recorded for NM-2011 (Fig 6). However, the highest NAR was noted for genotype NM-20-21 and the least for NM-51 (Fig 7).

**Fig 6:** Crop growth rate of various mungbean genotypes at various growth stages as affected by Zn fertilization.

**Fig 7:** Net assimilation rate of various mungbean genotypes at various growth stages as affected by Zn fertilization.

### Yield and yield components

Zinc application at 10 kg ha^-1^ significantly (p≤0.05) improved the plant height (1.58–10.70%), number of reproductive branches per plant (9.49–26.67%) and number of vegetative branches (20.75–30.38%) of all mungbean genotypes (Table 1). Genotypes NM-51 and NM-92 observed the highest plant height (87.00 and 86.00 cm, respectively) because of more response to Zn availability. Likewise, genotype NM-92 performed superior regarding the number of reproductive (45.00) and vegetative branches (38.00) with Zn fertilization (Table 1).

**Table 1:** Effect of Zn application on plant height, number of vegetative branches per plant and number of reproductive branches per plant of different mungbean genotypes.

Genotypes	Plant height (cm)			Number of vegetative branches plant^-1^			Number of reproductive branches plant^-1^		
	0 kg	10 kg	Means	0 kg	10 kg	Means	0 kg	10 kg	Means
**NM-28**	74.66 g	81.33 d	78.00 E	33.00 hi	41.00 c	37.00 D	30.66 fg	36.33 bc	33.50 AB
**NM-2011**	67.00 k	71.66 h	69.33 I	27.33 n	33.00 hi	30.16 H	25.00 l	27.66 j	26.33 H
**NM-2006**	77.00 f	82.66 c	79.83 D	32.00 ij	40.33 c	36.16 E	31.00 f	37.00 b	34.00 A
**NM-13-1**	65.00 l	68.33 ij	66.66 J	30.00 kl	39.00 d	34.50 F	27.66 j	31.00 f	29.33 E
**NM-51**	81.66 cd	87.00 a	84.33 A	34.66 fg	43.00 b	38.83 B	31.00 f	35.66 c	33.33 B
**NM-54**	71.66 h	79.33 e	75.50 F	34.00 gh	44.33 a	39.16 B	29.00 i	33.33 d	31.16 C
**NM-92**	80.00 e	86.00 a	83.00 B	35.33 ef	45.00 a	40.16 A	30.00 gh	38.00 a	34.00 A
**NM-19-19**	63.00 m	64.00 lm	63.50 L	26.00 o	32.00 ij	29.00 I	26.00 k	28.66 i	27.33 G
**NM-20-21**	63.33 m	67.33 jk	65.33 K	28.33 mn	36.00 e	32.16 G	24.66 l	27.00 j	25.83 H
**NM-121-25**	68.66 i	72.66 h	70.66 H	29.33 lm	35.66 ef	32.50 G	28.66 i	32.00 e	30.33 D
**7006**	79.33 e	84.33 b	81.83 C	33.66 gh	42.33 b	38.00 C	29.33 hi	34.00 d	31.66 C
**7008**	69.33 i	76.00 f	72.66 G	31.00 jk	38.66 d	34.83 F	27.33 j	30.00 gh	28.66 F
**Means**	71.72 B	76.72 A		31.22 B	39.19 A		28.36 B	32.55 A	

Means not sharing the same letters within a column differ significantly from each other at 5% level of probability. Plant height LSD value at 5% for genotypes (G) = 0.92; Zn = 0.37; G × Zn = 1.30, number of vegetative branches per plant LSD value at 5% for genotypes (G) = 0.72; Zn = 0.29; G × Zn = 1.03, number of reproductive branches per plant LSD value at 5% for genotypes (G) = 0.50; Zn = 0.20; G × Zn = 0.71.

Zinc fertilization enhanced all yield components, including the number of grains, pod length and grain weight per pod for all mungbean genotypes as compared to control (Table 2). The genotypes NM-92 and NM-51 recorded a higher number of grains per pod, pod length and grain weight per pod, whereas genotypes 7008 and NM-20-21 recorded the lowest values of these traits (Table 2).

**Table 2:** Effect of Zn application on pod length, number of grains per pod and grain weight per pod of different mungbean genotypes.

Genotypes	Pod length (cm)			Number of grains per pod			Grain weight per pod (g)		
	0 kg	10 kg	Means	0 kg	10 kg	Means	0 kg	10 kg	Means
**NM-28**	8.02 j	8.46 e	8.24 D	9.00 fg	9.66 de	9.33 CD	0.42 hi	0.47 c-e	0.44 DE
**NM-2011**	6.73 r	7.77 m	7.25 I	7.33 Kk	7.66 jk	7.50 GH	0.36 kl	0.40 ij	0.38 G
**NM-2006**	8.33 f	8.62 c	8.47 B	9.00 fg	10.33 bc	9.66 BC	0.46 d-g	0.49 bc	0.48 bc
**NM-13-1**	7.23 q	7.86 kl	7.54 H	7.33 k	8.33 hi	7.83 G	0.37 kl	0.44 gh	0.40 F
**NM-51**	8.37 f	8.74 b	8.56 A	9.33 ef	10.66 ab	10.00 AB	0.47 c-f	0.50 ab	0.49 B
**NM-54**	7.83 l	8.19 h	8.01 E	8.66 gh	9.33 ef	9.00 DE	0.40 ij	0.46 e-g	0.43 E
**NM-92**	8.27 g	8.84 a	8.55 A	9.33 ef	11.00 a	10.16 A	0.49 b-d	0.53 a	0.51 A
**NM-19-19**	7.43 p	7.90 k	7.66 G	7.66 jk	9.00 fg	8.33 F	0.38 jk	0.42 hi	0.40 F
**NM-20-21**	6.32 s	7.72 n	7.02 J	6.66 l	7.33 k	7.00 I	0.34 lm	0.37 kl	0.36 H
**NM-121-25**	7.63 o	8.12 i	7.88 F	8.33 hi	9.00 fg	8.66 EF	0.38 jk	0.42 hi	0.40 F
**7006**	8.14 i	8.52 d	8.33 C	8.66 gh	10.00 cd	9.33 CD	0.44 f-h	0.48 b-e	0.46 CD
**7008**	6.11 t	7.69 n	6.90 K	6.33 l	8.00 ij	7.16 HI	0.33 m	0.35 lm	0.34 H
**Mean**	7.53 B	8.20 A		8.13 B	9.19 A		0.40 B	0.44 A	

Means not sharing the same letters within a column differ significantly from each other at 5% level of probability, Pod length LSD value at 5% for genotypes (G) = 0.03; Zn = 0.01; G × Zn = 0.04, number of grains per pod LSD value at 5% for genotypes (G) = 0.41; Zn = 0.16; G × Zn = 0.58, grain weight per pod LSD value at 5% for genotypes (G) = 0.01; Zn = 0.008; G × Zn = 0.02.

Zinc fertilization enhanced 1000-grain weight, grain yield and biological yield of all mungbean genotypes than control (Table 3). Likewise, genotype NM-51 produced the highest grain and biological yields, whereas NM-2011 had the lowest grain and biological yields (Table 3). Zinc application enhanced chlorophyll contents and harvest index of all genotypes as compared to control (Table 4). Genotypes NM-5, 7006 and NM-2006 remained superior regarding chlorophyll contents and harvest index, respectively. Likewise, genotype NM-19-19 performed poorly for chlorophyll contents and was statistically similar to NM-13-1 (Table 4).

**Table 3:** Effect of Zn application on 1000-grain weight, and grain and biological yields of different mungbean genotypes.

Genotypes	1000-grain weight (g)			Grain yield (kg ha^-1^)			Biological yield (kg ha^-1^)		
	0 kg	10 kg	Means	0 kg	10 kg	Means	0 kg	10 kg	Means
**NM-28**	46.33 h	50.00 de	48.16 D	726.5 n	999.9 d	863.2 E	3084.9 k	3841.0 e	3463.0 F
**NM-2011**	38.33 no	41.66 l	40.00 H	439.2 x	536.5 u	487.9 L	2030.3 v	2614.1 p	2322.2 K
**NM-2006**	47.00 gh	54.00 c	50.50 C	798.8 j	1051.8 c	925.3 C	3045.0 l	3952.2 d	3498.6 D
**NM-13-1**	39.66 mn	44.33 ij	42.00 G	517.1 v	679.3 p	598.2 J	2524.2 r	2995.9 m	2760.1 H
**NM-51**	46.66 gh	56.33 b	51.50 B	904.4 f	1462.3 a	1183.4A	3501.9 g	4746.4 a	4124.1 A
**NM-54**	42.33 kl	45.66 hi	44.00 F	811.8 i	927.6 e	869.7 D	3218.3 i	4118.1 c	3668.2 C
**NM-92**	48.00 fg	58.00 a	53.00 A	875.7 g	1216.7 b	1046.2B	3382.4 h	4549.0 b	3965.7 B
**NM-19-19**	40.00 m	45.66 hi	42.83 G	660.7 q	790.5 k	725.6 G	2373.2 u	2941.2 n	2657.2 J
**NM-20-21**	37.66 op	38.66 m-o	38.16 I	579.2 t	745.0 m	662.1 I	2408.4 t	2913.4 o	2660.9 J
**NM-121-25**	43.00 jkl	49.00 ef	46.00 E	605.1 s	758.0 l	681.6 H	2575.2 q	3053.4 l	2814.3 G
**7006**	43.66 jk	51.33 d	47.50 D	708.0 o	860.9 h	784.4 F	3148.8 j	3802.1 f	3475.5 E
**7008**	36.33 p	38.00 o	37.16 J	485.6 w	622.7 r	554.1 K	2467.7 s	3002.4 m	2735.1 I
**Means**	42.41 B	47.72 A		676.0 B	887.6 A		2813.4 B	3544.1 A	

Means not sharing the same letters within a column differ significantly from each other at 5% level of probability, 1000 grain weight LSD value at 5% for genotypes (G) = 0.96; Zn = 0.39; G × Zn = 1.36, grain yield LSD value at 5% for genotypes (G) = 4.16; Zn = 1.69; G × Zn = 5.88, biological yield LSD value at 5% for genotypes (G) = 7.29; Zn = 2.97; G × Zn = 10.31.

**Table 4:** Effect of Zn application on chlorophyll contents, harvest index and grain Zn contents of different mungbean genotypes.

Genotypes	Chlorophyll Contents (SPAD value)			Harvest index (%)			Grain Zn contents (mg kg^-1^)		
	0 kg	10 kg	Means	0 kg	10 kg	Means	0 kg	10 kg	Means
**NM-28**	40.23 mn	42.30 k	41.26 G	23.56 j	26.00 de	24.78 D	22.50 p	46.40 e	34.45 F
**NM-2011**	40.66 lm	49.43 b	45.05 C	21.60 l	20.53 m	21.06 I	20.30 q	29.30 mn	24.80 I
**NM-2006**	44.50 hi	48.30 c	46.40 A	26.23 d	26.60 c	26.41 C	45.60 e	64.23 a	54.91 A
**NM-13-1**	36.03 q	41.43 kl	38.73 J	20.46 m	22.66 k	21.56 H	15.50 s	18.53 r	17.01 J
**NM-51**	41.50 kl	46.43 ef	43.96 D	25.83 e	30.80 a	28.31 A	25.93 o	36.33 ij	31.13 H
**NM-54**	37.06 p	47.26 de	42.16 EF	25.20 g	22.50 k	23.85 F	31.23 l	49.50 d	40.36 D
**NM-92**	44.20 ij	47.40 cd	45.80 AB	25.90 e	26.73 c	26.31 C	43.06 f	60.20 b	51.63 B
**NM-19-19**	35.70 q	43.40 j	39.55 I	27.83 b	26.86 c	27.35 B	28.00 n	32.13 l	30.06 H
**NM-20-21**	40.10 mn	40.50 m	40.30 H	24.03 i	25.53 f	24.78 D	40.26 gh	52.40 c	46.33 C
**NM-121-25**	39.46 n	45.63 fg	42.55 E	23.50 j	24.83 h	24.16 E	37.20 i	41.26 g	39.23 D
**7006**	40.20 mn	50.43 a	45.31 BC	22.50 k	22.66 k	22.58 G	30.83 lm	34.13 k	32.48 G
**7008**	38.23 o	45.20 gh	41.71 FG	19.66 n	20.73 m	20.20 J	35.20 jk	39.36 h	37.28 E
**Means**	39.82 B	45.64 A		23.86 B	24.70 A		31.30 B	41.98 A	

Means not sharing the same letters within a column differ significantly from each other at 5% level of probability, chlorophyll contents LSD value at 5% for genotypes (G) = 0.65; Zn = 0.26; G × Zn = 0.92, harvest index LSD value at 5% for genotypes (G) = 0.19; Zn = 0.07; G × Zn = 0.26, grain Zn contents LSD value at 5% for genotypes (G) = 1.24; Zn = 0.50; G × Zn = 1.75.

### Grain Zn-biofortification

Significant variability was observed among mungbean genotypes for grain Zn contents, which ranged from 15 to 45 mg kg^-1^. Zinc application improved grain Zn contents of all genotypes, which ranged from 19 to 64 mg kg^-1^ (Table 4). The response of the genotypes was not the same for Zn biofortification. Zinc contents of the genotype NM-28 improved by 24 mg kg^-1^, which was the highest, while in contrast Zn contents in genotype NM-31-1 improved by 3 mg kg^-1^ only which was the lowest (Table 4).

## Discussion

This study indicated that mungbean genotypes with Zn application had better allometric traits (i.e., root length, number of lateral roots, LAI, CGR, LAD and NAR) as compared to no-Zn fertilization (Figs 1–6). Better allometric traits with Zn-fertilization might be attributed to the association of Zn with the synthesis of nucleic acid, protein, lipids, carbohydrates, nitrogen metabolism, photosynthesis, cell division and other related cell processes [36–38]. Better root growth and improved number of lateral roots might be attributed to involvement of Zn in the stimulation of several metabolic enzymes in the root cells [39], which promote cell division and elongation [11, 12, 27–29]. Zinc fertilization improves the resistance against abiotic stresses by improving the root morphology and physiology [40], which ultimately enhances root growth.

Better seedling growth and grain yield of mungbean genotypes grown under Zn application might be attributed to the contribution of Zn in physiological processes during plant development [41, 42], protein synthesis, photosynthesis [43], nitrogen use efficiency and resistance to abiotic stresses [44]. This increase in growth might be due to existence of Zn, which triggers certain enzymes responsible for the cell processes leading to taller plants [1, 23, 45]. These findings are also in line with Dashadi [46] who concluded that Zn dynamically takes part in auxin production, which increases the cell size and quantity; thus, enhancing plant height. Kabir et al. [47] reported that Zn-deficiency negatively affected biomass production, cellular integrity and chlorophyll synthesis in tomato. Likewise, Saboor et al. [48] reported that combination of arbuscular mycorrhizal fungi and biofertilizer-based Zn improved growth and yield of maize.

Harvest index and grain yield are products of growth and development. As discussed above, Zn application improves growth and development by enhancing nitrogen use efficiency, protein synthesis, antioxidant mechanism, root development and plant morphological traits, which ultimately result in higher grain yield [24]. Several scientists have concluded that Zn application at different levels in mungbean crops significantly enhanced grain yield [11, 12, 27–29]. Usman [49] reported that the highest number of grains per pod, 1000-grain weight, and grain and biological yields were achieved with Zn-fertilization. Along with yield, Zn-biofortification was another major objective of this study. Results revealed that soil application of Zn improved Zn-biofortification of mungbean grains, but a huge variation was observed in diverse germplasm for bioavailability of Zn contents. Genotypes differed for Zn uptake due to their diverse genomic makeup and regulation of enzymes related to Zn uptake and assimilation [50–52]. Nair [50] reviewed the genetic diversity of mungbean for iron and Zn and reported a significant potential of improving through biofortification as he found 20–40 g Zn concentration kg^-1^ for dry mungbean seed and the nearly same range was also observed in our study under control conditions and was further improved to 64 g kg^-1^. Singh [20] mapped 15 QTLs through composite interval mapping that were linked with Zn concentration on chromosome numbers 4, 6, 7, 11 of mungbean. They further proposed the use of SSR markers associated with identified QTLs for Zn-biofortification in mungbean. The response of the genotypes to soil-applied Zn also varied and some genotypes respond more regarding the bioavailability of Zn contents in the seed. Therefore, genotypes with high bioavailable Zn and better capacity to uptake soil-applied Zn should be used in breeding programs for sustainable Zn-biofortification.

## Conclusions

Zinc fertilization improved yield and grain Zn contents with significant differences among tested genotypes during the current study. Genotypes NM-92 and NM-51 performed better for grain yield; however, NM-2006 and NM-28 proved better for grain Zn-biofortification. Therefore, the genotypes NM-28 and NM-2006 could be used in breeding programs for improvement in grain Zn-concentration. Nonetheless, all available genotypes in the country should be screened for their Zn-biofortification potential.
